# Immunosuppressive functions of melanoma cell-derived exosomes in plasma of melanoma patients

**DOI:** 10.3389/fcell.2022.1080925

**Published:** 2023-01-06

**Authors:** Theresa L. Whiteside

**Affiliations:** Depts of Pathology, Immunology and Otolaryngology, University of Pittsburgh School of Medicine and UPMC Hillman Cancer Center, Pittsburgh, PA, United States

**Keywords:** melanoma, small extracellular vesicles, exosomes, melanoma cell-derived exosomes (MTEX), immune capture, immune suppression

## Abstract

Tumor-derived exosomes (TEX) are a subset of small extracellular vesicles (sEV) present in all body fluids of patients with cancer. In plasma of patients with metastatic melanoma, numbers of exosomes produced by melanoma cells called MTEX are elevated. To study the role of MTEX in melanoma progression, immunoaffinity-based separation of MTEX from total plasma exosomes was performed. The surface of MTEX was decorated by various checkpoint inhibitory proteins, and upon coincubation with immune recipient cells, MTEX suppressed anti-tumor functions of these cells. MTEX emerge as a major mechanism of immune suppression in melanoma and thus might play a role in promoting melanoma progression.

## Introduction

Extracellular vesicles (EVs) are produced and released by all cells. However, stressed cells, including cancer cells, produce an excess of EVs, and plasma of cancer patients is enriched in circulating tumor cell-derived vesicles called TEX. The main function of EVs is intercellular communication, which involves the transfer of information between cells, especially cells distantly located from one another. EVs are heterogenous and vary broadly in size, cellular origin, biogenesis and molecular/genetic cargos they carry (Whiteside, 2017). TEX are a subset of circulating EVs with unique characteristics that set them apart from other vesicles (Czystowska-Kuzmicz and Whiteside, 2021). Specifically, TEX originate from the late endosomes/multi-vesicular bodies (MVBs) in tumor cells and are released into extracellular space upon fusion of MVBs with the cell membrane. They are small vesicles sized at 30–150nm, and their surface topography as well as the lumen content resemble those of parent tumor cells (Czystowska-Kuzmicz and Whiteside, 2021). The current EV nomenclature places TEX in the category of small EVs (sEV) or exosomes (Thery et al., 2018), and it emphasizes their distinction from larger microvesicles (MVs) ranging in size from 200 to 500 nm and from much larger apoptotic bodies based not only on the vesicle size but also distinct biogenesis. Melanoma cell-derived TEX (MTEX) circulate freely and cross the BBB as well as all organ barriers (Banks et al., 2022). Upon contact with the cell membrane of recipient cells, MTEX enter into the cytosol, engaging various mechanisms that facilitate their entry, including receptor/ligand signaling, membrane fusion, integrin-mediated uptake, opsonization, endocytosis or phagocytosis (Mulcahy et al., 2014). The vesicle entry results in transcriptional and molecular changes in the recipient cell. These changes reflect the ability of MTEX to re-program functions of recipient cells (Czystowska-Kuzmicz and Whiteside, 2021).

This commentary discusses the interactions of TEX derived from melanoma cells (MTEX) with immune cells and describes the consequences of MTEX-mediated transfer of information from the tumor to immune cells. The impact of the MTEX-T cell crosstalk is emphasized as an example of cancer-driven functional reprogramming that promotes melanoma progression by inducing dysfunction of immune cells, especially CD8^+^ effector T-cell.

### MTEX isolation from melanoma patients’ plasma

For the study described here (Sharma et al., 2020), the banked plasma specimens from patients with metastatic melanoma and healthy donors (HD) were obtained from the U. of Pittsburgh Melanoma SPORE Bank (IRB #991206). All study participants signed an informed consent form. The banked specimens were annotated and were randomly selected for the studies described here. Thawed plasma samples were pre-cleared by centrifugation and were ultrafiltered prior to size exclusion chromatography (SEC) as previously described (Hong et al., 2016). Small extracellular vesicles (sEV) were eluted in the void volume with PBS and harvested in fraction #4. Following concentration with 100,000 MWCO Vivaspin 500 centrifugal concentrators, protein levels of vesicles were measured using a BCA protein assay kit. The vesicle size and particle numbers were verified using qNano or NanoSite. Transmission electron microscopy (TEM) was used to visualize the vesicles. The sEV isolated from melanoma plasma had the vesicular morphology, a mean size of 90–110 nm and were positive for tetraspanins (CD63, CD81), TSG101 and ALIX, but were negative for the cytosolic proteins, calnexin and grp94 in western blots. TAM images of sEV obtained from a melanoma patient’s plasma were similar in the morphology and size to sEV isolated from plasma of patients and HDs (Figure 1). Total sEV protein levels were higher in patients than in HDs: mean 76 μg/ml vs. 54 μg/ml (Figure 2A) and were not significantly different in melanoma patients with no evident disease (NED) or active metastatic disease at blood draw for this study (Sharma et al., 2020). Total plasma-derived sEV in the SEC fraction #4 were used for the separation of MTEX from non-malignant cell-derived vesicles, non-MTEX.

**FIGURE 1:** Transmission electron microscopy images of sEV from a healthy donor’s plasma (left) and from a melanoma patient’s plasma (right).

**FIGURE 2:** Protein levels in total plasma exosomes of melanoma patients or HDs and in isolated MTEX. In **(A)**, total exosome protein (TEP) levels in plasma of HDs or melanoma patients. In **(B)**, the total MTEX/TEP ratio for all patients vs. patients with NED or with progressive disease following oncological therapy. In **(C)**, protein levels in MTEX obtained from plasma of NED patients or melanoma patients with metastases (i.e., progressive disease following oncological.

MTEX isolation from total plasma exosomes was performed by immune capture using the melanoma cell-specific monoclonal Abs provided by Dr. Soldano Ferrone (Harvard U.) Anti-CSPG4 mAbs (clones 763.64 and 225.28) recognize an epitope of CSPG4 (also known as the high molecular weight melanoma associated antigen) present on melanoma cells but not on any other non-malignant cells or tissues as determined by immunostaining and previously reported (Campoli et al., 2004). The capture mAb (763.64) was biotinylated, and MTEX captured by the biotinylated mAb harvested on streptavidin-charged magnetic beads as described (Sharma et al., 2018). The non-captured vesicles were recaptured using biotinylated anti-CD63 mAb and streptavidin beads. Both fractions, MTEX and non-MTEX, were studied by on-bead flow cytometry for their protein profiles (Theodoraki et al., 2021), and the detected protein expression levels were calculated as Relative Fluorescence Intensity (RFI) values equal to the ratio of MFI detection mAb/MFI isotype control. TEM of isolated MTEX and non-MTEX showed vesicles with morphology similar to that of total plasma EVs, although the MTEX size was somewhat smaller than that of non-MTEX. The protein content of isolated MTEX ranged from 20 to 60µg/ml and was no different for melanoma patients with NED vs. patients with progressive disease (PD) after oncologic therapy (Figure 1B). The MTEX/total sEV protein (TEP) ratio was also not different for these two patient groups (Figure 1C). Among 12 melanoma patients, MTEX represented 23%–66% of total plasma sEV (Sharma et al., 2020). This may appear as a very high proportion of recovered MTEX, and it contrasts with the scarce data for the recovery of cancer TEX from plasma reported in the literature. In one study of patients with NSCLC, anti-EpCAM Abs were used to capture TEX, and their recovery ranged from 0.5%–11% of total plasma sEVs(Yoh et al., 2021). In other studies, TEX were identified based on the TEX associated gene expression profiles (Wu et al., 2021), with recoveries that were very low (Vitale et al., 2021) or by microfluidics based capture on chips, where co-expression levels of tumor-associated antigens (TAA) present on TEX were high, but TEX recovery was not evaluated (Zhao et al., 2016; Yu et al., 2021). The broad frequency range of MTEX recovered from plasma seen in our study suggests that the MTEX/non-MTEX ratios vary with disease activity, as two of the patients in our small cohort with the highest MTEX recovery had advanced ocular melanoma with pulmonary and liver metastases.

Immunocapture of MTEX with anti-CSPG4 mAb proved to be highly effective, largely due to its specificity for the melanoma cells/exosomes and its high binding avidity. As such, it has been repeatedly used in our studies of MTEX. Specificity of the immunocapture for MTEX was verified by demonstrating that MTEX isolated from various melanoma cell lines showed the presence of CSPPG4 on all sEVs albeit at various expression levels; only MTEX isolated from plasma were CSPG4+, while non-MTEX were CSPG4 (-); sEV obtained from plasma of HDs were CSPG4 (-) and only MTEX were highly enriched in melanoma-associated antigens (MAA), TYRP2, Melan A, Gp100, VLA4; only non-MTEX were CD3^+^, while MTEX were CD3 (−). When MTEX were added to vesicles obtained from HDs plasma in spiking experiments, immune capture recovered all CSPG4+ vesicles, while the non-captured fraction was CSPG4 (−).

### Protein profiles of MTEX and non-MTEX

On-bead flow cytometry of MTEX and non-MTEX was performed as previously described (Theodoraki et al., 2021) to evaluate their surface protein profiles, primarily looking at the expression levels of immunoregulatory proteins. Table 1 and Table 2 list RFI values for immunosuppressive and immunostimulatory surface proteins on MTEX isolated from 12 patients with melanoma. By adding individual RFI values for all surface proteins carried on MTEX, we calculated the suppressor and stimulatory RFI scores for each patient (Table 1). The sum of the suppressor or stimulatory scores gave the mean RFI scores for all 12 patients. The same set of data was obtained for all paired non-MTEX fractions (data not shown). Although the same immunoregulatory proteins were detectable in MTEX and non-MTEX, the mean RFI score for *immunosuppressive* proteins was significantly higher (*p* = 0.03) for MTEX (15.3) than for non-MTEX (11.7). The mean RFI score for *immunostimulatory* proteins was significantly lower (*p* = 0.002) for MTEX (8.8) than for non-MTEX (16.2). Both suppressive and stimulatory scores for non-MTEX were similar to those calculated for sEV of HDs. We also calculated the stimulatory/suppressor ratio for MTEX, which was significantly lower (*p* = 0.001) than the ratio for non-MTEX or for sEV of HDs at 0.6, 1.4 and 2.2, respectively. In aggregate, the quantitative flow cytometry data indicated that MTEX were significantly enriched in immunosuppressive surface proteins, while non-MTEX largely carried immunostimulatory surface proteins. This observation indicated that MTEX are more likely to mediate suppression of immune cells than non-MTEX or sEV from plasma of HDs.

**TABLE 1:** Immunosuppressive proteins in MTEX^a^.

Patient	Supp RFI Score^b^	PD1	PDL-1	CD39	CD73	Fas	FasL	LAP-TGFβ	TRAIL	CTLA-4
1	16.8	3.3	4	1	1.2	4	1.8	4	3.8	1
2	13.4	1.6	1	1.8	2.4	2	2.2	1	3.8	1.2
3	13	1.1	2.5	3	1	1	2	1	1	2.5
4	20.3	8	1.6	1.1	1	4.8	7.2	1.8	6	1.6
5	15.2	2.8	1.8	2	1	2.3	2.8	3	3.6	1
6	10.8	5.9	1	1	2.9	2.3	2.3	1	1	1.6
7	19.9	2	1.2	1.5	1	2.8	4.8	4.8	4	2.6
8	16.7	6.8	3.9	1.4	1	2.6	4.4	3.7	1.3	1
9	17.1	6.2	4.2	1.4	1	1.3	2.4	3.8	2.5	1.8
10	9.8	5.8	1.3	1.3	1	5	2.4	1	1	1.8
11	15.5	6.5	1.4	2.7	2.2	2.5	2.8	1.8	3.6	1
12	15.2	6.1	1	3.4	1.4	2.4	2.3	1.3	3.2	2.6

^a^ Proteins detected on the surface of MTEX by on-bead flow cytometry.

^b^ Supp RFI Score = the sum of PD1, PD-L1, CD39, CD73, Fas, FasL, LAP-TGFβ, and CTLA4.

The mean RFI Score for immunosuppressive proteins in MTEX, 15.3.

**TABLE 2:** Immunostimulatory proteins in MTEX.^a^.

Patient	Stim RFI score^a^	CD40	CD4OL	CD80	OX40	OX4OL
1	14.4	1	1	3	4	5.4
2	5.3	1	1.1	1	1.1	1.1
3	6.2	1	1.1	1	1.1	2
4	12	1	4.2	1	3.5	2.3
5	6.4	1	1	1	1	2.4
6	6	1	1.1	1	1.4	1.5
7	10.7	1	1	1	3.8	3.9
8	6.6	1	1.2	1.2	1.2	2
9	7.2	1	1	1.2	1.9	2.1
10	14.6	1	2.2	1.2	3	7.2
11	8.9	1	1.1	1	3.7	2.1
12	7.2	1	1	1	1.7	2.5

^a^ Stim RFI score = the sum of CD40, CD40L, CD80, OX40 and OX40L.

The mean RFI Score for immunostimulatory proteins in MTEX, 8.8.

## Immunosuppressive functions of MTEX and non-MTEX

Immunoregulatory activities of MTEX, non-MTEX and sEV of HDs were evaluated in co-incubation experiments with human primary immune cells (Figure 3). The following functional assays were performed: CD69 protein downregulation on the surface of T cells, changes in CD69 mRNA transcripts in T cells, NF-κB activation in CD8^+^ T cells, CSFE-based proliferation of CD8^+^ T cells, apoptosis of CD8^+^ T cells and NKG2D down-regulation on the surface of NK cells. Utilizing primary *in vitro* activated CD8+T cells or natural killer (NK) cells as vesicle recipient cells in co-incubation experiments, we compared inhibitory effects of MTEX and non-MTEX on the above listed immune cell functions. MTEX captured on beads were used in these assays, while non-MTEX and sEV of HDs were in solution. The presence of beads alone or beads coated with biotinylated CSPG4 capture mAbs did not interfere with the functional assays (data not shown). Table 3 summarizes results of these assays.

**FIGURE 3:** Measurement of TEX-induced phenotypic and functional changes in T cells following their co-incubation with TEX or sEV from cancer plasma. Following co-incubation at optimized doses for different time periods depending on the assay, T cells were tested for the vesicle uptake or entry into the cytosol or for changes in the surface protein profile, in growth and apoptosis levels or in mRNA transcription. Vertical stipled lines indicate that inhibitors of the T cell-TEX crosstalk can be used to block T cell-TEX interactions.

**TABLE 3:** Results of coincubation assays of the isolated vesicles with immune cells ^a^.

Assay	MTEX	Non-MTEX	HD sEV
% T-cell with CD69 expression (flow cytometry)	45% (*p* = 0.0005)	90%	90%
CD8^+^T-cell NF-κB activation (p65 nuclear trans-location by confocal microscopy	Yes	No	No
%CD8^+^T-cell Proliferation (CSFE)	25% (*p* = 0.0005)	85%	75%
%CD8^+^T-cell Apoptosis (Annexin/PI binding)	83% (*p* = 0.0005)	20%	25%
%NK cells with surface NKG2D expression	70% (*p* = 0.001)	95%	98%
CD8^+^T-cell Changes in CD69 transcripts (RT-PCR)	Decrease	No change	No change

^a^ Primary human T cells and NK cells were co-incubated with paired MTEX, and non-MTEX, or with sEV from HDs (6 h for apoptosis, NKG2D assays or RT-PCR; 72 h for CSFE assays and 30min for NF-κB activation). The data are median values of results obtained in experiments performed in triplicates for 12 patients with metastatic melanoma (Sharma et al., 2020).

Coincubation of the isolated vesicles with human primary T cells or NK cells led to significant inhibition of activation, proliferation and survival of the immune cells interacting with MTEX but not of cells coincubated with non-MTEX or sEV obtained from plasma of HDs. The data in Table 3 are median values for inhibitory functions of the vesicles from 12 patients with metastatic melanoma. The ranges of inhibitory activity of MTEX and non-MTEX varied broadly among the patients. While non-MTEX paralleled the functional behavior of sEV of HDs in all assays, in some patients, non-MTEX showed mild inhibitory activity (Sharma et al., 2020). This observation suggested that non-MTEX, derived from plasma of melanoma patients, were not functionally identical with sEV of HDs.

We previously reported that TEX co-incubated for 6 h with human primary T cells were not readily internalized but remained at the T-cell surface for 15–30min (Muller et al., 2017). This observation suggested that both CD69 (an activation antigen) downregulation in T cells and apoptosis of CD8^+^ T cells measured at 6 h of coincubation with MTEX may be initiated by cell surface signaling events, which then translate into cellular alterations in T cells. Indeed, using RT-PCR we showed that MTEX, but not non-MTEX, induced downregulation of CD69 mRNA transcripts in CD8^+^ T cells following 6 h coincubation. Also, a 30 min coincubation of CD8^+^ T cells with MTEX induced translocation of the NF-κB subunit p65 to the nucleus of a T cells, confirming activation of the NF-κB pathway and surface signaling by MTEX, which leads to downregulation of the CD69 expression level. It has been reported that the normally pro-inflammatory NF-κB pathway leads to cellular apoptosis in cancer, where stress due to genetic, metabolic or environmental factors drives the cell damage responses (Janssens et al., 2014; Cao et al., 2016). Vesicles in all three fractions, MTEX, non-MTEX and HD sEV, induced vesicle dose-dependent apoptosis in activated CD8^+^T cells; however, MTEX induced significantly higher apoptosis than non-MTEX, which was only partially blocked by neutralizing anti-Fas (ZB4) mAbs. MTEX induced down-regulation of NKG2D (a cytolysis activating antigen) expression levels on the surface of NK cells, and thus inhibited NK cell activity. Preliminary experiments in which we attempted to interfere with the inhibitory signaling of MTEX by preincubation with neutralizing Abs to surface proteins on the MTEX surface showed only a partial and never complete inhibition of apoptosis. Also, the correlations linking the observed functional inhibition with expression of any single inhibitory protein on the MTEX surface were not significant, except for apoptosis, which was only partly blocked with anti-Fas mAb. The experiments with neutralizing mAbs suggested that not any one but rather several simultaneously delivered receptor-ligand signals might be responsible for MTEX mediated apoptosis in activated human primary CD8^+^T cells (Sharma P, et al., 2020).

Interestingly, MTEX mediate suppression of immune functions that exclusively target anti-tumor immune responses and do not appear to interfere with responses to infections. Such selective suppression of anti-tumor immunity is seen in most patients with malignancies (Whiteside, 2006; Chen and Mellman, 2013), but its severity varies broadly among patients and may relate to disease progression. Thus, patients with melanoma have variously depressed anti-tumor immunity but appear to respond normally to viral or bacterial antigens, except for patients with advanced metastatic disease, whose immune system may be generally compromised.

### MTEX and non-MTEX protein profiles *versus* their functional attributes

Functional changes induced in recipient immune cells by MTEX and non-MTEX were correlated with the protein profiles of these vesicles. Total exosome protein (TEP) levels in plasma correlated with the MTEX immunosuppressive score (*p* = 0.002, *r* = 0.79), linking the high TEP levels with the enrichment in suppressive MTEX. Thus, apoptosis correlated with the MTEX/TEP ratio (*p* = 0.01, *r* = 0.68). The RFI scores for FasL and TRAIL in MTEX were significantly elevated relative to non-MTEX, accounting for high MTEX-driven apoptosis. The stim/supp ratio correlated positively with the immuno-stimulatory score (*p* = 0.006, *r* = 0.74). Unexpectedly, apoptosis mediated by non-MTEX was inversely correlated with the stim/supp ratio (*p* = 0.007, *r* = -0.75) and with the immunostimulatory score (*p* = 0.009, *r* = -0.72). Non-MTEX -induced proliferation of T cells positively correlated with their immunostimulatory score (*p* = 0.04, *r* = 0.59). In aggregate, these and other correlations linking immune activities of MTEX and non-MTEX with their phenotypic characteristics showed that: i) MTEX had superior immune suppressor activity *vis a vis* non-MTEX; ii) the stimulatory/inhibitory vesicle activities were dependent on the surface profile of immunoregulatory proteins in MTEX and non-MTEX; and iii) MTEX and non-MTEX abilities to alter functions of immune receptor cells depended on the stim/suppr protein ratios in these vesicles.

### MTEX and non-MTEX profiles and patients’ clinicopathological data

The group of patients we evaluated consisted of 12 individuals (6 males and six females) aged 32–82 years, previously treated with oncological therapies. Five of these patients had no evident disease (NED) and seven had progressive disease at the time of blood draw for this study. We attempted to explore associations of the observed characteristics of MTEX and non-MTEX with disease status or activity in this small cohort of melanoma patients. While the study was not powered for a formal correlative assessment, it provided several potentially important insights. While MTEX-mediated apoptosis of CD8^+^T cells did not correlate with disease status or stage at diagnosis, the non-MTEX ability to induce apoptosis associated with disease stage (*p* = 0.04, r = 0.61). This was an unexpected observation, which suggests that non-MTEX might potentially serve as a correlate of disease progression in future studies. We also observed a significant inverse correlation between of the stim/supp ratio with disease stage (*p* = 0.0007, r = -0.83). This suggests that the stim/supp ratio might be more informative about disease progression than individual regulatory protein expression in the vesicular profile. In this study, with the exception of an inverse correlation between disease status and PD-L1 expression levels in MTEX (*p* = 0.03, r = -0.62), no other regulatory proteins on the MTEX surface correlated with disease status or activity.

## Concluding remarks

It has been reported that TEX isolated from supernatants of tumor cell lines carry on their surface immunosuppressive ligands, FasL, TRAIL and immunosuppressive proteins such as TGF-β or CD39/CD73, and suppress functions of immune cells *in vitro* and *in vivo* in tumor-bearing mice (Ludwig et al., 2018; Razzo et al., 2020). Recent studies confirm that the surface of sEV (exosomes) isolated from plasma of melanoma patients is decorated by immunosuppressive proteins, including PD-L1 (Chen et al., 2018; Cordonnier et al., 2020). The cellular source of these immunosuppressive vesicles in plasma has remained unknown, however. Here, we considered the evidence for a major role played by MTEX isolated from plasma of patients with melanoma in suppression of immune cell functions. The immunoaffinity-based separation of MTEX from the non-malignant cell-derived exosomes (non-MTEX) in melanoma patients’ plasma allowed for the analysis and comparison of molecular cargos of MTEX and non-MTEX and for establishing MTEX as the main source of immunosuppressive signals delivered to recipient immune cells. MTEX are abundant in plasma of melanoma patients, and in patients with metastatic melanoma, MTEX might represent a majority of circulating vesicles. In this context, MTEX emerge as a major immunosuppressive mechanism that promotes melanoma escape from the host immune system. Our data are in agreement with other reports on tumor-promoting attributes of melanoma-derived EVs (Peinado et al., 2012; Gyukity-Sebestyen et al., 2019; Bollard et al., 2020; Amor Lopez et al., 2021).

To support this conclusion, we showed that the short-term (6 h) coincubation of MTEX with activated effector (CD8^+^T and NK cells) reduced CD69 expression levels and initiated apoptosis in CD8^+^T-cell or reduced NKG2D expression in NK cells contributing to the attenuation of NK activity (Hong et al., 2014). These results suggest that signaling *via* MTEX-associated surface proteins is sufficient for eliciting changes in the phenotype or function of recipient T or NK cells. The downregulation of CD69 expression on the T-cell surface was followed by changes in CD69 mRNA transcripts in recipient T cells, indicating that signals delivered by MTEX resulted in transcriptional activation. Further, a 30min coincubation of MTEX with CD8+T cells induced activation of the NF-κB pathway, as evidenced by the translocation of p65 to the nucleus of the recipient cells. These results clearly implicate MTEX in functional reprogramming of normal human effector cells. Interestingly, non-MTEX isolated from peripheral blood of patients with melanoma, but not sEV from plasma of HDs, also downregulated functions of immune cells, albeit much less effectively than MTEX. This observation indicates that non-malignant cells in patients with melanoma may be subverted by the tumor to also produce immunosuppressive vesicles, contributing to melanoma progression. The presented evidence for MTEX as drivers of molecular and transcriptional changes in effector immune cells of patients with melanoma calls for additional studies of MTEX in larger cohorts of patients to better define their role in melanoma progression and confirm their clinical significance.
